This article has been retracted.

# Nestin Regulates Autophagy‐Dependent Ferroptosis Mediated Skeletal Muscle Atrophy by Ubiquitinating MAP 1LC3B

**DOI:** 10.1002/jcsm.13779

**Published:** 2025-04-04

**Authors:** Shunshun Han, Xiyu Zhao, Chunlin Yu, Can Cui, Yao Zhang, Qing Zhu, Mohan Qiu, Chaowu Yang, Huadong Yin

**Affiliations:** ^1^ College of Animal Science and Technology Key Laboratory of Livestock and Poultry Multi‐Omics, Ministry of Agriculture and Rural Affairs Sichuan Agricultural University Chengdu Sichuan China; ^2^ Farm Animal Genetic Resources Exploration and Innovation Key Laboratory of Sichuan Province Sichuan Agricultural University Chengdu Sichuan China; ^3^ Animal Breeding and Genetics Key Laboratory of Sichuan Province Sichuan Animal Science Academy Chengdu China

**Keywords:** autophagy, ferroptosis, MAP 1LC3B, nestin, skeletal muscle atrophy

## Abstract

**Background:**

Programmed cell death plays a critical role in skeletal muscle atrophy. Ferroptosis, an iron‐dependent form of programmed cell death driven by lipid peroxidation, has been implicated in various diseases, but its role in skeletal muscle atrophy remains unclear.

**Methods:**

Ferroptosis in skeletal muscle atrophy was investigated using two models: dexamethasone (Dex)‐induced atrophy (*n* = 6 independent cell cultures per group) and simulated microgravity (*n* = 6 mice per group). Conditional Nestin knockout (KO) mice were generated using CRISPR/Cas9 (*n* = 6–8 mice per group), with wild‐type (WT) controls (*n* = 6–8). Phenotypic analyses included histopathology (HE staining), functional assessments (muscle strength, weight analysis, treadmill), and dystrophy evaluation (dystrophin staining). Molecular analyses involved flow cytometry, ELISA, transmission electron microscopy, PI staining, and IP/MS to delineate Nestin‐regulated ferroptosis pathways in skeletal muscle atrophy.

**Results:**

Ferroptosis was significantly activated in both atrophy models, with a 2.5‐fold increase in lipid peroxidation (*p* < 0.01), a 2‐fold accumulation of Fe^2+^ (*p* < 0.01) and a 50% reduction in Nestin expression (*p* < 0.001). Nestin KO mice exhibited exacerbated muscle atrophy, showing a 40% decrease in muscle weight (*p* < 0.01) and a 30% reduction in muscle strength (*p* < 0.05) compared to WT mice. Nestin overexpression mitigated Dex‐induced ferroptosis, reducing lipid peroxidation by 40%, decreasing Fe^2+^ accumulation by 50% (*p* < 0.01), and improving muscle function by 30% (*p* < 0.05). Mechanistically, Nestin interacted with MAP 1LC3B (LC3B) to catalyse LC3B polyubiquitination at lysine‐51, reducing LC3B availability for autophagy and inhibiting autophagy flux by 60% (*p* < 0.01), leading to a 50% reduction in ferroptosis (*p* < 0.001).

**Conclusions:**

Our study identifies Nestin as a critical regulator of ferroptosis‐autophagy crosstalk in skeletal muscle atrophy. Targeting Nestin‐LC3B ubiquitination may offer novel therapeutic strategies for preventing muscle wasting in diseases such as cachexia and sarcopenia.

## 1 Introduction

Skeletal muscle atrophy is a clinical condition characterized by muscular weakness and loss of muscle mass [1]. Skeletal muscle atrophy is caused by multifarious conditions, including long‐term inactivity, aging, diabetes, cancer and cachexia [2]. Patients with muscle atrophy develop disabilities and become unable to perform essential self‐care tasks, which can result in morbidity and mortality. An imbalance in protein synthesis and degradation leads to muscle atrophy, and the accelerated breakdown of protein significantly affects muscle quality and functionality [3]. A series of genes, known as ‘atrogenes’ (atrophy‐related genes) have been discovered to control complex biochemical and transcriptional processes that affect various forms of muscle atrophy [4]. As atrogenes are implicated in the muscle atrophy pathophysiology, Trim63 (MuRF1) and MAFbx (Atrogin‐1) show greatly increases in diverse muscle atrophy forms in mice or humans [5]. Studies have revealed that programmed cell death (PCD), such as autophagy, apoptosis, and necrosis, are crucial for maintaining and restoring muscle integrity through muscle‐specific activation of atrogenes (Trim63 and MAFbx) [6].

Iron‐dependent death, also known as ferroptosis, is a novel form of PCD [7]. However, its role in muscle atrophy remains unknown. Ferroptosis, unlike apoptosis, autophagy, and necrosis, is characterized by a decrease in GSH levels, the inactivation of GPX4, and ultimately the accumulation of iron‐dependent lipid peroxides [8]. Ferroptosis is believed to be closely related to the pathogenesis of numerous medical conditions, including cancer [9], liver fibrosis [10], spinal cord injury [11], inflammation [12], and cardiovascular disease [8]. However, the pathogenicity of ferroptosis in skeletal muscle has not been revealed. Thus, identifying novel ferroptosis regulators is crucial for the therapy of skeletal muscle atrophy and other disorders.

Nestin is an intermediate filament protein that belongs to the cytoskeletal family, which facilitates cell mechanical stability [13]. Nestin plays a crucial role in the organization of myofibrils, differentiation of myotubes, and maintenance of the contractile apparatus [14]. Moreover, Nestin knockdown confers neural progenitor cells susceptible to exogenous oxidant stress‐induced cell death, indicating that Nestin plays a crucial role in determining survival under oxidative stress [15]. Wang et al. discovered that Nestin enhances the generation of antioxidant enzymes through the Keap1‐Nrf2 feedback loop and regulates redox homeostasis in non‐small cell lung cancer [16]. The Keap1‐Nrf2 feedback loop is a crucial pathway that regulates ferroptosis [17]. Therefore, these reports have shown that Nestin may be involved in the ferroptosis signalling pathway associated with skeletal muscle atrophy. Further investigation is required to ascertain the potential involvement of Nestin in the ferroptosis signalling pathway, thereby regulating skeletal muscle atrophy and weakness.

In this study, we elucidated the molecular mechanism of ferroptosis in skeletal muscle atrophy. We found a strong correlation between ferroptosis and skeletal muscle atrophy, with Nestin being identified as a crucial factor in the occurrence of ferroptosis events. Skeletal muscle atrophy induces downregulation of Nestin, which antagonizes autophagy by promoting LC3B ubiquitination and accelerating iron‐dependent lipid peroxide accumulation, eventually resulting in ferroptosis. Our findings suggest that Nestin plays a crucial role in the pathogenesis of ferroptosis‐induced skeletal muscle atrophy and represents a promising therapeutic target for its treatment.

## 2 Methods

### 2.1 Animals

Animal protocols were approved by the Animal Ethics Committee of Sichuan Agricultural University, and strict adherence to the guidelines of the Experimental Animal Welfare and Animal Experimentation Ethics Committee of Sichuan Agricultural University was followed (Approval number: SAULAB‐2019‐04‐25). Skeletal muscle conditional Nestin knockout mice were generated using CRISPR/Cas9 approach at Biocytogen Pharmaceuticals Co. Ltd. (Beijing, China). Exons 1–4 of Nestin were inserted into the flanking LoxP sites to produce two LoxP sites. These were subsequently electroporated into C57BL/6 J mouse embryonic stem cells to produce Nestin^*flox/flox*^ mice. Then, Nestin^*flox/flox*^ mice were crossed with MYF5‐Cre mice to generate Nestin mice with a conditional knockout (cKO) of skeletal muscle. To induce the muscle atrophy model, Dex or PBS was intraperitoneally injected at a dosage of 25 mg/kg/per. All mice were sacrificed with sodium pentobarbital after one week. All of the mice utilized in this study were genetically C57BL/6J aged between 8 and 10 weeks.

### 2.2 Measurements of Muscle Force and Muscle Weight

Under anaesthesia, six male and six female mice aged 8 weeks from Nes KO and control groups were humanely euthanized. SOL, EDL, GAS, and TA were quickly collected and weighed electronically. The methodology for quantifying muscular strength was as previously delineate [18]. In summary, the 305B muscle lever system (Aurora Scientific, Aurora, Ontario, Canada) was used to test the contractile function of the gastrocnemius muscle in anaesthetised mice. Electrical stimulation of the sciatic nerve elicited muscular contraction. By dividing torque by the length of the lever arm, force generated by the plantar flexor muscles was estimated.

### 2.3 Reactive Oxygen Species (ROS) Assay

Briefly, the cells were expanded in 12‐well plates for 24 h and then treated with 20 μM DCFH‐DA dye (Sigma‐Aldrich) for 30 min at 37°C. The cells were trypsinized (Sigma‐Aldrich) to obtain a cell suspension, which was then washed with PBS for three times. The levels of ROS were analysed using a flow cytometer.

### 2.4 Lipid Peroxidation, GSH, and Iron Assay

C2C12 cells were cultured in 12‐well plates. After specific treatment, the cell lysate was obtained by centrifugation. Then, according to the manufacturer's instructions, MDA (cat. no. ab118970, Abcam) or 4‐NHE (cat. no. ab238538, Abcam) lipid peroxidation detection kit was used to measure the quantity of lipid peroxidation products in the cell lysates. The concentration of GSH in cell lysates was measured using a GSH assay kit (cat. no. CS0260; Sigma‐Aldrich). An iron assay kit (cat. no. ab83366, Abcam) was used to measure the concentration of iron in the cell lysate.

### 2.5 Plasmid constructs

Plasmids GFP‐LC3B, HA‐Ub, Nestin‐Flag were provided by Sangon Biotech (Shanghai, China). GFP‐LC3B mutants (K5R, K8R, K30R, K39R, K42R, K51R, K65R, K103R, K122R) were generated using PCR or the Q5® Site‐Directed Mutagenesis Kit (Biolabs, Beijing, China).

### 2.6 Statistical Analysis

All of the results are presented as means ± S.D. Student's paired *t*‐test was used to compare the means of two groups. More than two groups were compared using one‐way analysis of variance (ANOVA). The Least Significant Difference test was used for post hoc comparisons of group differences when the ANOVA was significant. GraphPad Prism 6.0 Software was used for all statistical calculations. Statistical significance was defined as a *p*‐value less than 0.05. ‘n.s.’ refers to differences that are not statistically significant.

## 3 Results

### 3.1 Ferroptosis Occurs in Skeletal Muscle Atrophy and Nestin Expression Decreases Both In Vivo and In Vitro

To investigate the role of ferroptosis in skeletal muscle atrophy, C2C12 cells were treated with the synthetic glucocorticoid Dex or ferroptosis activator erastin. As expected, the average diameter of the myotubes significantly decreased after Dex treatment or Erastin (Figure S1A). Additionally, the expression of atrogenes Trime63 and MAFbx were significantly increased following treatment with Dex or erastin (Figure S1B). Similar to erastin treatment, Dex treatment resulted in a significant decrease in cell viability as revealed by CCK8 and PI staining (Figure 1A). After Dex treatment, GSH levels dramatically decreased, while MDA levels, GSSG, iron content, and lipid peroxidation increased considerably (Figure 1B). Western blot analysis revealed a significant downregulation in the expression of FTH1 and GPX4, while the protein levels of ACSL4 were significantly upregulated after Dex treatment (Figure 1C). Then, through the mechanical unloading and disuse, we utilized the tail suspension model to lead to hind limb atrophy (Figure S1C,D). The results confirmed that ferroptosis plays an important role in skeletal muscle atrophy both in vitro and in vivo (Figure S1E). Then, we treated myotubes with lip‐1 after Dex treatment to investigate the role of ferroptosis in skeletal muscle atrophy, it was observed that ferroptosis was inhibited after lip‐1 treatment (Figure 1D). Furthermore, Trim63 and MAFbx expression were dramatically downregulated after lip‐1 treatment, and significantly enhanced the fusion rate of myoblasts into myotubes (Figure 1E). These findings suggest that the prevention of ferroptosis may alleviate skeletal muscle atrophy.

**FIGURE 1:** Ferroptosis occurs in skeletal muscle atrophy, and the expression of Nestin is decreased. (A) CCK8 and PI staining was used to detect cell viability in C2C12 cells after incubation with Dex (10 μM) for 1, 2, 3 days, or with Eratin (5 μM) for 24 h in differentiation medium. DAPI was used as counterstain the nuclei (blue). Scale bars, 100 μm (*n* = 6). (B) The intracellular levels of GSH, MDA, 4‐HNE, iron content and ROS were detected after incubation with Dex for 1, 2, 3 days, or with Eratin (5 μM) for 24 h in differentiation medium (*n* = 6). (C) Western blot was used to measure the protein expression levels of ACSL4, FTH1, and GPX4 in C2C12 cells after incubated with Dex for 1, 2, 3 days or Eratin (5 μM) for 24 h in differentiation medium. Tubulin as loading control (*n* = 3). (D) C2C12 cells were pre‐treated with Dex for 24 h, either with or without lip‐1 treatment. PI staining or ELISA assays was detected the intracellular levels of GSH, MDA, 4‐HNE, iron content, ROS or cell survival were detected by (*n* = 6). (E) C2C12 cells were pre‐treated with Dex for 24 h, either with or without lip‐1 treatment. qPCR analysis was conducted to measure the mRNA expression levels of Trim63 and MAFbx (*n* = 3). Immunocytochemical staining of myosin heavy chain (MyHC) using a pan‐myosin heavy chain antibody (Red). DAPI was used to counterstain the nuclei (blue). Scale bar, 100 μm (*n* = 3). (F) Western blot measured the protein expression levels of Nestin in C2C12 cells after incubated with Dex for 1, 2, 3 days, or with Eratin for 24 h in differentiation medium (*n* = 3). qPCR analysis the mRNA expression levels of Nestin (*n* = 3). Data are means ± SD. *p < 0.05; **p < 0.01; ***p < 0.001.

Interestingly, Nestin expression was significantly downregulated both in vivo and in vitro during muscle atrophy (Figure 1F and Figure S1F). Based upon these findings we speculated Nestin's involvement in the ferroptosis pathway, leading to skeletal muscle atrophy.

### 3.2 Nestin Knockout Results in Muscle Atrophy and Weakness in Mice

Next, we detected the expression pattern of Nestin in different mouse tissues and found that Nestin was highly expressed in skeletal muscle (Figure S2A). Then, we investigated the effect of Nestin on skeletal muscle atrophy in vivo. Consequently, we generated Nestin skeletal muscle‐conditional knockout (cKO) mice (Figure S2B,C). Morphometric observations revealed that the weight of GAS, SOL, EDL, and TA in the Nestin cKO mice was considerably lower than those of control mice (Figure 2A). HE staining revealed a reduced cross‐sectional area in the Nestin cKO mice (Figure 2B and S2D,E). Moreover, immunofluorescence staining revealed a 53% decrease in muscle fibre cross‐sectional area in Nestin knockout mice compared to control within the gastrocnemius muscle (*p* < 0.05)(Figure 2C). The Nestin knockout mice consistently had lower body weight than the control mice at 2 and 5 months of age, indicating reduced muscle tissue in Nestin‐deficient mice (Figure S2F). Next, we investigated whether muscular atrophy in live animals was followed by muscle strength loss. In both male and female Nestin knockout mice, the absolute skeletal muscle force was dramatically decreased (Figure 2D). Even after normalizing the absolute force of the muscle mass, the specific force produced remained 1.2–1.5 folds lower (*p* < 0.05) (Figure 2E). The Nestin cKO mice exhibited a reduction in running time and distance during the forced treadmill test, suggesting impaired muscle performance (Figure 2F). The findings suggest that Nestin is essential in preventing skeletal muscle weakness and atrophy.

**FIGURE 2:** Morphological and functional changes in *Nestin* cKO mice. (A) Representative graphs of GAS, SOL, EDL and TA in control and Nestin *cKO* mice (*n* = 6). (B) H&E staining was used to examine the size of GAS myofibers and various features of muscle deterioration in control and Nestin cKO mice (*n* = 6). Scale bar, 50 μm. (C) The cross‐sectional area of GAS muscle fibres in control and Nestin cKO mice were stained by immunofluorescence with anti‐dystrophy antibody, and measured the average cross‐sectional area of GAS in control and Nestin cKO mice (*n* = 6). (D) Force measurements were performed on GAS during tetanic contraction in control and Nestin cKO mice, and the absolute tetanic force is normalized to the muscle weight at aged 2 months or 5 months in control and Nestin cKO mice (*n* = 6). (F) The running length of mice forced to run on the treadmill until exhaustion was used to measure muscle performance in control and Nestin cKO mice (*n* = 6). Data are means ± SD. *p < 0.05; **p < 0.01; ***p < 0.001.

To validate the findings in vitro, C2C12 myoblasts were transfected with Ad‐shNestin to silence or with Ad‐Nestin to overexpress Nestin expression (Figure S3A). We found that Nestin negatively regulates the mRNA and protein expression of MAFbx and Trim63 (Figure S3B,C). Additionally, the myotube fusion index significantly decreased in Nestin‐silenced cells, while overexpressing Nestin enhanced it (Figure S3D). To further investigate Nestin's role in muscle atrophy, we induced atrophy in differentiated myotubes by treating C2C12 cells with Dex. The expression levels of two ‘atrogenes’ were significantly increased in Nestin‐silenced cells after Dex treatment, while their expression levels were decreased with Nestin overexpression (Figure S3E). Furthermore, Dex‐treated Nestin‐deficient cells exhibited reduced myotube fusion index, which was rescued by Nestin overexpression (Figure S3F). These findings suggest that Nestin plays a crucial role in regulating muscle atrophy and hypertrophy by modulating of the atrogenic system.

### 3.3 Nestin Regulates Skeletal Muscle Atrophy by Mediating Ferroptosis

To explore the effect of Nestin on skeletal muscle atrophy, we cultured the primary myoblasts from the gastrocnemius muscles of control and Nestin cKO mice (Figure 3A). The mRNA and protein levels of ACSL4 in Nestin cKO myoblast cells increased by 1.5‐fold (*p* < 0.01), while the expression of FTH1 and GPX4 was downregulated by 2‐fold (*p* < 0.01) (Figure 3B). Further evidence that Nestin knockout‐induced ferroptosis events (Figure 3C,D). After 48 h of culture in differentiation media, we conducted RNA‐Seq analysis on control and Nestin cKO myotubes. The results revealed significant alterations in the expression of genes associated with myogenesis, autophagy, and iron homeostasis in Nestin‐deficient myotubes. The KEGG pathway analysis showed that differentially expressed genes (DEGs) were clearly associated with autophagy, P53, mTOR, and ferroptosis pathways, all of which are closely related to iron homeostasis (Figure 3E). And GO functional annotation analysis of DEGs identified genes involved in the muscle system process, striated muscle contraction, and response to iron ions (Figure 3F). These results suggest that Nestin may impact skeletal muscle development by regulating iron homeostasis.

**FIGURE 3:** Nestin knockout promotes ferroptosis, and liproxstatin‐1 ameliorates ferroptosis to promote functional recovery after Nestin deficiency. (A) Western blot analysed of Nestin protein expression levels in control and Nestin cKO myoblast cells. Tubulin as loading control (*n* = 3). (B) The mRNA or protein level of ACSL4, FTH1, and GPX4 were assessed by qPCR or western blot in control and Nestin cKO myoblast cells. Tubulin as loading control (*n* = 3). (C) CCK8 was used to detect cell viability in control and Nestin cKO myoblast cells, and the values of intracellular GSH, MDA, 4‐HNE, iron content and ROS levels were measured in control and Nestin cKO myoblast cells (*n* = 6). (D) Mitochondrial state was assessed in Ctrl and Nestin cKO myoblast cells using Mito‐Tracker Red CMXRos. Scale bars, 50 μm (*n* = 6). (E) Grading clustering and heatmap analysis were performed to compare the expression of ferroptosis‐ and autophagy‐related genes in control and Nestin cKO myoblast cells (*n* = 3). (F) The top 11 enhanced pathways in control compared with Nestin cKO myoblast cells were revealed by KEGG analysis of the RNA‐seq data. And functional annotation was analysed against down‐regulated genes in control compared with Nestin cKO cells. Data are means ± SD. *p < 0.05; **p < 0.01; ***p < 0.001.

To determine whether Nestin deletion directly contributes to ferroptosis, we treated Nestin cKO myoblast cells with ferroptosis activator or inhibitor. We found that Nes cKO cells were significantly more susceptible to cell death than WT cells when treated with a ferroptosis activator or inhibitor (Figure S4A–F). Additionally, lip‐1 treatment reduced ferroptosis induced by Nestin knockout, while erastin treatment increased ferroptosis events (Figure S5A–D). Further, lip‐1 treatment restored the ability of myoblast differentiation into myotubes, while the fusion index of myotubes in erastin‐treated Nestin cKO myoblast cells was reduced by approximately 20% (Figure S5E). Additionally, qPCR analysis revealed that Nestin deletion could promote the expression of the muscle atrogenes by triggering ferroptosis events (Figure S5F).

We injected lip‐1 into Nestin cKO mice to investigate if Nestin knockout triggers skeletal muscle atrophy via the ferroptosis pathway. The results showed that lip‐1 could significantly alleviate ferroptosis caused by the knockout of Nestin (Figure S6A,B). Morphology analysis revealed that treatment with lip‐1 significantly increased the weight of GAS, SOL, EDL, and TA muscles in Nestin cKO mice (Figure S6C), as well as resulted in larger cross‐sectional areas of muscle fibres (*p* < 0.01) (Figure S6D). Further measurements demonstrated that lip‐1 treatment improved both force and muscle performance in forced treadmill running tests for Nestin cKO mice (Figure S6E). And lip‐1 treatment significantly inhibited the expression levels of MAFbx and Trim63 in Nestin cKO mice (Figure S6F). These data collectively indicate that Nestin deletion triggers ferroptosis, causing skeletal muscle atrophy.

### 3.4 Nestin Knockdown Promotes Ferroptosis In Vitro

To further determine the role of Nestin in iron homeostasis, C2C12 cells were pre‐treated with Ad‐shNestin or Ad‐Nestin to silence or express Nestin, respectively. Western blotting revealed that Ad‐Nestin markedly reduced Nestin expression levels in Dex‐treated C2C12 cells or untreated cells, while Ad‐Nestin dramatically increased its expression (Figure 4A). Silencing Nestin exacerbated the ferroptosis event, and this effect persisted even when the cells were treated with Dex or erastin. Furthermore, overexpression of Nestin can mitigate the occurrence of ferroptosis induced by Dex or erastin (Figure 4B–D). Then, the results of CCK8 and PI assays demonstrated that overexpression of Nestin partially reversed the inhibition of cell activity, conversely knockdown of Nestin further increased cellular sensitivity to death (Figure 4E,F). These findings suggest that Nestin depletion increases susceptibility to ferroptosis events in C2C12 cells.

**FIGURE 4:** Nestin negatively regulates ferroptosis in vitro. C2C12 cells were treated with Ad‐shCtrl, Ad‐shNestin, Ad‐Ctrl or Ad‐Nesin and incubated with Dex (10 μM) for 24 h or Erastin (5 μM) for 24 h. (A) The protein level of Nestin was assessed by western blot analysis. Tubulin as loading control (*n* = 3). (B) The values of intracellular GSH, MDA, 4‐HNE, iron content and ROS levels were detected (*n* = 6). (C) Mitochondrial state was assessed using Mito‐Tracker Red CMXRos. Scale bars, 50 μm (*n* = 6). (D) The mRNA or protein expression levels of ACSL4, FTH1, and GPX4 were measured by qPCR or western blot. Tubulin as loading control (*n* = 3). (E) Cell viability was detected by CCK8 under Erastin or Dex treatment conditions (*n* = 6). (F) C2C12 cells were treated with Erastin or dexamethasone at the indicated time. PI staining was used to detect cell survival in C2C12 cells transfected with Ad‐shCtrl, Ad‐shNestin, Ad‐Ctrl or Ad‐Nesin (*n* = 6). Data are means ± SD. *p < 0.05; **p < 0.01; ***p < 0.001.

### 3.5 Nestin Deletion‐Mediated Ferroptosis is Associated With Autophagy Activation

Ferroptosis has been described as a type of autophagy‐dependent programmed cell death [19]. Thus, we elucidated whether Nestin could affect skeletal muscle atrophy through autophagy‐mediated ferroptosis. Western blotting demonstrated that the overexpression of Nestin prevented LC3‐II expression levels, whereas silencing of Nestin increased LC3‐II expression (Figure 5A). We investigated the protein expressions of three autophagy marker genes: ATG5, ATG7 and Beclin1. The results showed significant upregulation in Nestin‐silenced cells and marked downregulation in Nestin‐overexpression cells (Figure 5B). Immunofluorescence staining confirmed that Nestin could drastically reduce Beclin1 protein expression (Figure 5C). We transfected C2C12 cells with mRFP‐GFP‐LC3 adenovirus to measure autophagy flux. Confocal microscopy revealed a 1.8‐fold (*p* < 0.01) increase in autophagosomes in Nestin‐silenced cells and a 1.6‐fold (*p* < 0.01) decrease in autophagosomes in Nestin‐overexpressing cells (Figure 5D). Finally, TEM showed a 1.7‐fold (*p* < 0.01) increase in autophagosomes silenced by Nestin, while the number of autophagosomes treated with Ad‐Nestin significantly decreased by 2‐fold (*p* < 0.01) (Figure 5E). To examine the role of autophagy inhibition by Nestin in ferroptosis using either CQ or ATG5 knockdown to inhibit autophagy (Figure S7A,B). We found that Nestin silencing‐induced ferroptosis may be partially reversed by inhibiting autophagy through CQ or knockdown of ATG5 (Figure S7C–F). These data validate the hypothesis that autophagy activation triggers ferroptosis induced by Nestin deletion.

**FIGURE 5:** Ferroptosis suppressed by Nestin is related with autophagy inactivation. (A) Western blot analysed LC3B protein expression levels in C2C12 cells after transfected with Ad‐shCtrl, Ad‐shNestin, Ad‐Ctrl or Ad‐Nesin for 24 h. Tubulin as loading control (*n* = 3). (B) Western blot analysed the protein of autophagy‐related gene (ATG5, ATG7 and Beclin1) after transfected with Ad‐shCtrl, Ad‐shNestin, Ad‐Ctrl or Ad‐Nesin for 24 h. Tubulin as loading control (*n* = 3). (C) The immunofluorescence intensity of the Beclin1 protein was detected by Beclin1 antibody and DAPI (nuclei) in Ad‐shCtrl, Ad‐shNestin, Ad‐Ctrl or Ad‐Nesin cells. Scare bar, 200 μm (*n* = 3). (D) C2C12 cell were transfected with mRFP‐GFP‐LC3 adenovirus for 24 h, and confocal imaging was used to count the number of autophagosomes in Ad‐shCtrl, Ad‐shNestin, Ad‐Ctrl or Ad‐Nesin cells (*n* = 3). (E) Cells were transfected with Ad‐shCtrl, Ad‐shNestin, Ad‐Ctrl, or Ad‐Nesin for 24 h, and analysed using transmission electron microscopy to identify autophagosomes (*n* = 3). Data are means ± SD. *p < 0.05; **p < 0.01; ***p < 0.001.

### 3.6 Nestin Interacts With LC3B Antagonizing Autophagy System

To study the molecular mechanism of Nestin‐mediated regulation of autophagy‐induced ferroptosis, we utilized IP/MS analysis and found that LC3B was identified as a potential Nestin‐interacting protein (Figure 6A). Co‐IP assay showed that endogenous Nestin directly interacts with LC3B. However, neither control IgG nor Nrf2 (which can bind Nestin and control ferroptosis) precipitated (Figure 6B). Meanwhile, we performed a Co‐IP with GFP and Flag‐Nestin‐tagged proteins in HEK 293 T cells. As expected, exogenous GFP‐labelled LC3B interacted with Flag‐labelled Nestin (Figure 6C).

**FIGURE 6:** Nestin regulates autophagy‐mediated ferroptosis through interaction with LC3B. (A) IP/MS was used to detect the interacting peptide between Nestin and LC3B. (B) LC3B and Nestin were examined by immunoblotting using the designated antibodies, and endogenous levels in myoblasts cell lysate protein binding were tested by immunoprecipitation with anti‐Nestin or anti‐LC3B (*n* = 3). (C) HEK 293T cells were transfected with Flag‐labelled Nestin and GFP‐labelled LC3B. The lysate from these cells was immunoprecipitated with anti‐Flag or anti‐GFP, followed by immunoblotting with anti‐GFP‐LC3B or anti‐Flag‐Nestin (*n* = 3). (D) Schematic representations of wild‐type and deletion mutants of Flag‐tagged Nestin are shown. (E) GFP‐tagged LC3B was co‐expressed with several truncated Flag‐tagged Nestin proteins in HEK293T cells. Protein G beads and anti‐GFP antibody were used for the immunoprecipitation process (*n* = 3). (F) pcDNA3.1, Flag‐Nestin, or Nestin (N1478‐1864) was transfected into Nestin‐knockdown cells using the appropriate manner. Immunoblotting was used to examine the expression levels of LC3B, ACSL4, FTH1, and GPX4 (*n* = 3). Data are means ± SD. *p < 0.05; **p < 0.01; ***p < 0.001.

To determine how Nestin binds to LC3B, full‐length and truncated Flag‐labelled Nestin fragments were constructed and co‐expressed with GFP‐labelled LC3B in HEK 293T cells (Figure 6D). Co‐IP analysis revealed that GFP‐LC3B specifically interacted with the full length (N1–1864) and fragments containing amino acids (N701–1864 and N1478–1864) within the C‐terminal tail of Flag‐Nestin, suggesting that Nestin fragments N1478–1864 can bind to LC3B (Figure 6E). Furthermore, we observed that the N1478–1864 fragment of Nestin protein was sufficient to reverse Nestin knockdown‐induced ferroptosis by binding with LC3B (Figure 6F). These findings suggest a direct binding between Nestin and LC3B, indicating their crucial role in maintaining autophagy balance during ferroptosis.

### 3.7 Nestin Promotes the Ubiquitination and Degradation of LC3B

Furthermore, we investigated the impact of Nestin on LC3B expression in C2C12 cells. Nestin deficiency increased LC3B protein levels in cells treated with or without erastin or Dex, but had no effect on LC3B mRNA levels compared to the control (Figure S8A–F). This suggests that Nestin post‐transcriptionally regulates the stability of LC3B protein. Then, we treated with proteasome inhibitor MG132, which reversed the decreases in LC3B protein levels induced by Nestin overexpression (Figure 7A). Moreover, the half‐life of LC3B was memorably decreased in the Nestin‐overexpression cells in the presence of CHX, but not in the Nestin (C111A)‐overexpression cells (Figure 7B). Co‐IP assay demonstrated that Nestin overexpression significantly increased ubiquitinated LC3B protein levels, while Nestin silencing or Nestin (C111A) mutants inhibited ubiquitination (Figure 7C). To determine the site of Nestin‐mediated LC3B ubiquitination, we observed that there are 10 lysine ubiquitination sites in the amino acid sequence of LC3B (Figure 7D). The 10 lysines of LC3B were mutated to arginine, preventing their conjugation with ubiquitin. The results showed that the K51R mutants were not ubiquitinated, indicating that lysine 51 was the main site for LC3B ubiquitination (Figure 7E). We constructed several LC3B mutants and found that LC3B‐K51R, with arginine replacing lysine 51, was not ubiquitinated by Nestin (Figure 7F), indicating that Nestin targets lysine‐51 for ubiquitination on LC3B.

**FIGURE 7:** Nestin promotes LC3B ubiquitination and degradation. (A) Examining the levels of the LC3B and Nestin proteins in C2C12 cells transfected with Ad‐Nestin, either with or without the proteasome inhibitor MG132 (*n* = 3). (B) LC3B and Nestin were analysed in HEK 293 T cells transfected with Nestin‐Flag or Nestin (C111A) mutant vector, and treated with cycloheximide (CHX, 200 μg/mL) for a specified time (*n* = 3). (C) Exogenous LC3B ubiquitination tests were performed in the lysates of HEK 293 T cells transduced with Nestin shRNA, Nestin overexpression, or the Nestin Mutation vector, and the immunocomplexes were assessed by western blotting (*n* = 3). (D) The sequence of mouse LC3B is shown, with lysine residues highlighted in red. (E) HEK 293T cells were transfected with a plasmid encoding WT and a series of mutant LC3B constructs, as well as HA‐Ub. Anti‐GFP immunoblotting was performed, followed by HA and anti‐GFP immunoblotting (*n* = 3). (F) The wild‐type or each of the LC3B mutations, tagged with GFP, were transfected into HEK293T cells. Anti‐GFP antibody was used to immunoprecipitate exogenous LC3B or each of the LC3B mutants, and an immunoblot was used to test for ubiquitination (*n* = 3). Data are means ± SD. *p < 0.05; **p < 0.01; ***p < 0.001.

### 3.8 LC3B Knockdown Inhibits the Ferroptosis Induced by Nestin Knockdown

To determine whether decreased autophagy alleviates Nestin knockdown‐induced ferroptosis, Ad‐shLC3B was used to inhibit autophagy, whereas Ad‐LC3B was used to activate it in the Dex‐treated or untreated cells (Figure S9A). Therefore, we investigated the impact of LC3B overexpression or silencing on Nestin‐silenced‐induced ferroptosis events. Detailed information about each group's in vitro experiment is provided in Figure S9B. LC3B knockdown completely abolished ferroptosis events in control or Nestin‐deficient cells. In contrast, LC3B overexpression significantly increased the occurrence of ferroptosis events compared to control and Nestin‐deficient cells (Figure S9C,D). In the presence of Ad‐shNestin, LC3B overexpression worsens the inhibitory effect on cell viability, while silencing LC3B significantly improves it (Figure S9E). Then, we found LC3B silencing significantly reduced the expression levels of Trim63 and MAFbx, which were promoted by Nestin deletion. The levels of Trim63 and MAFbx expression induced by Nestin deletion were further exacerbated with LC3B overexpression (Figure S9F). These results suggest that the absence of Nestin leads to ferroptosis via an autophagy‐dependent mechanism.

### 3.9 Nestin Deficiency Induces Ferroptosis and Limits Functional Recovery by Promoting LC3B Levels

Next, we investigated whether Nestin could directly target LC3B to induce ferroptosis and affect skeletal muscle atrophy. Mice were intramuscularly injected with AAV‐shNestin to generate skeletal muscle cell‐specific Nestin knockout mice. Then, AAV‐shLC3B and AAV‐LC3B were injected to explore their effects on skeletal muscle atrophy by ferroptosis events. The experimental group is described in detail in Figure 8A. Similar to the results of the aforementioned experiments in vitro, these results revealed that Nestin knockout promoted ferroptosis and resulted in a reduced in both muscle fibre cross‐sectional area and muscle mass compared with AAV‐Con (Figure 8B). The intramuscular injection of AAV‐shNes and AAV‐LC3B in mice further exacerbated ferroptosis, leading to inhibition of muscle fibre cross‐sectional area and muscle mass. However, AAV‐shLC3B injection significantly inhibited these adverse reactions and functional recovery of skeletal muscle (Figure 8C–E). Furthermore, LC3B overexpression induced ferroptosis, which further promoted skeletal muscle atrophy, and LC3B silencing could rescue skeletal muscle atrophy by inhibiting Nestin knockout‐induced ferroptosis events (Figure 8F). These findings suggest that Nestin maintains the skeletal muscle mass and structures by targeting LC3B‐mediated autophagy‐dependent ferroptosis.

**FIGURE 8:** Nestin knockdown promotes ferroptosis, thereby limiting functional recovery by increasing LC3B expression levels. (A) Information specific to the experimental group in this experiment. The generation of skeletal muscle cell‐specific Nestin knockout mice was achieved by intramuscular injection of AAV‐shNestin, followed by subsequent injections of AAV‐shLC3B or AAV‐LC3B. (B) qPCR and western blot analysis ACSL4, FTH1 and GPX4 mRNA and protein expression after injected with either AAV‐shLC3B or AAV‐LC3B in Nestin silenced or control skeletal muscle. Tubulin as loading control (*n* = 3). (C) H&E‐stained gastrocnemius muscles were investigated for morphological aberrations after injected with either AAV‐shLC3B or AAV‐LC3B in Nestin silenced or control skeletal muscle (*n* = 6). (D) After injecting either AAV‐shLC3B or AAV‐LC3B into Nestin‐silenced or control skeletal muscles, the cross‐sectional area of gastrocnemius muscle fibres was measured with anti‐dystrophy antibodies using immunofluorescence (*n* = 6). (E) The relative muscle weight of gastrocnemius (GC) or GC weight per body weight (BW) was measured after injected with either AAV‐shLC3B or AAV‐LC3B in Nestin silenced or control skeletal muscle (*n* = 6). (F) Western blot analysis was used to examine the protein expression of MAFbx and Trim63 after injection with either AAC‐shLC3B or AAV‐LC3B in Nestin silenced or control skeletal muscle. Tubulin as loading control (*n* = 3). Data are means ± SD. *p < 0.05; **p < 0.01; ***p < 0.001.

## 4 Discussion

Programmed cell death affects skeletal muscle development and homeostasis as a normal part of development or in response to pathological stimuli [20]. Dysregulation of PCD leads to muscle atrophy or sarcopenia [21]. In this study, we addressed a novel aspect that ferroptosis is related to the pathogenesis of skeletal muscle atrophy. In addition, the functional involvement of Nestin in controlling iron‐dependent cell death, which had not been reported previously, was demonstrated using loss‐of‐function and gain‐of‐function methods. Nestin deficiency activates autophagy by inhibiting the ubiquitination of LC3B, promoting the accumulation of iron‐dependent lipid peroxides and leading to iron‐dependent cell death. We offer a novel approach to improve treatment strategies for skeletal muscular dystrophy by targeting Nestin.

Iron is indispensable for the human body [22]. In almost all cells, iron plays an important role in the biological systems such as mitochondrial respiration, ATP production and the synthesis of haemoglobin [23]. In various physiological or pathological processes, iron also acts as a cofactor for many proteins and is involved in ferritin formation [24]. However, iron overload leads to the production of harmful hydroxyl radicals, which increase the levels of ROS and ultimately induce ferroptosis [25]. Studies have shown that iron overload negatively impacts skeletal muscle mass and function [26, 27]. DeRuisseau et al. observed a higher proportion of non‐heme iron in the skeletal muscles of elderly humans and aging rats, suggesting that increased iron concentration in the aging muscles is responsible for muscle mass loss [28]. Ikeda et al. discovered that iron overload triggers skeletal muscle atrophy by activating the Akt‐Forkhead box O3–E3 ubiquitin ligase‐dependent pathway [29]. This pathway is a key regulator of the atrophy‐related genes Trim63 and MAFbx [30]. In this study, we provide new evidence that ferroptosis induces skeletal muscle atrophy. Iron overload induces ferroptosis in muscle cells, disrupts lipid peroxide metabolism, and results in skeletal muscle atrophy. Therefore, ferroptosis, as well as autophagy and apoptosis, could possibly be crucial for the prevention management of muscular dystrophy.^S1, S2^

Several studies have demonstrated that Nestin strongly influences the growth of developing neurons,^S3^ initiates intracellular oxidative stress,^S4^ controls cell differentiation,^S5^ and promotes cancer progression.^S6^ Resting nestin‐positive progenitors can be activated under stress to participate in the maintenance and remodelling of various tissues, as well as to enhance the stress resistance of cells [31]. Wang et al. recently found that Nestin regulates cellular redox homeostasis by competitively binding to Keap1, thus preventing Keap1 from mediating Nrf2's ubiquitination degradation [32]. Nrf2 is a common marker gene of ferroptosis that governs the process via controlling GPX4 transcription, regulating glutathione production, and managing iron metabolism.^S7^ Therefore, Nestin may significantly affect ferroptosis by modulating iron metabolism‐related proteins. We observed a strong correlation between Nestin and muscle atrophy, and identified Nestin as playing a significant role in skeletal muscle atrophy through a newly defined iron‐dependent cell death mechanism. Furthermore, it was shown that Nestin regulates the transcription of a subset of atrophy‐related genes through the ferroptosis pathway to prevent muscle mass loss. As muscular atrophy is a dynamic process involving complex PCD, revealing the potential coordination mechanism of Nestin involved in cell death types may provide therapeutic targets for muscular atrophy.

Fe rroptosis has been associated with another physiological pathway, namely autophagy [33]. Autophagy is believed to be the upstream process that induces ferroptosis by controlling ROS production and iron metabolism [34]. Recent studies have shown that the occurrence of ferroptosis is dependent on autophagy, and many iron death regulators are considered potential factors in autophagy [19]. Hou et al. intracellular iron content and lipid peroxidation products were significantly reduced in human pancreatic cancer cell lines deficiency in either ATG5 or ATG7 [35]. Nestin deficiency was found to promote autophagosome formation and enhance autophagy flux, indicating a potential role of Nestin in inducing ferroptosis. Through IP/MS and immunoprecipitation assays, we found that Nestin's binding with LC3B protein antagonized the autophagy system. Studies have found that LC3B promotes the formation of autophagosomes by binding with ATG5/7 proteins during the autophagy process [36]. However, Nestin was not found to directly interact with ATG5/7 proteins in C2C12 cells (data not shown). Therefore, we hypothesize that Nestin prevents the formation of the ATG5/7–LC3B complex by destabilizing LC3B, ultimately blocking the autophagy pathway.

LC3B plays a pivotal role in the process of autophagy.^S8^ Under stress conditions, such as starvation or hypoxia, LC3B regulates autophagy and promotes cellular metabolic processes to maintain cell homeostasis.^S9^ Studies have reported that MAPLC3B‐mediated autophagy process enhances cell sensitivity to ferroptosis by promoting the degradation of ferritin [37]. Zhou et al. showed that ferroptosis is a form of cell death that depends on autophagy [19]. In skeletal muscles, Nestin deficiency may induce ferroptosis through LC3B‐mediated autophagy mechanisms. Studies investigating autophagy in muscle atrophy have revealed that excessive autophagy occurs during muscle degradation, which is accompanied by activation of the ubiquitin‐proteasome pathway.^S1^ In our study, we found that Nestin affects the stability of LC3B protein through post‐translational modifications. LC3B has been reported to be modified by E3 ubiquitin ligases, which regulate the ubiquitin protease system. Wu et al. found that the TRAF6‐catalysed K63 linkage of LC3B promoted autophagosome formation.^S10^ Kang et al. discovered that pVHL reduces the expression of LC3B by ubiquitinating it, thereby suppressing LC3B‐mediated autophagy.^S11^ We found Nestin interacts with LC3B to accelerate the ubiquitination of lysine 51 on the LC3B site, thereby reducing LC3B‐mediated autophagy, inhibiting ferroptosis, and maintaining skeletal muscle homeostasis. Lysine 51 of LC3B is a component of the hydrophobic pocket and is involved in recognizing the LIR motif of the autophagy receptor SQSTM1 [38]. SQSTM1 is a ubiquitin‐binding scaffold protein co‐localized with ubiquitinized protein aggregates in various diseases [39]. Therefore, the formation of the Nestin–LC3B complex may promote LC3B recognition by SQSTM1 and improve its ability to colocalize with ubiquitination substrates. These data indicate that Nestin maintains skeletal muscle atrophy and weakness through autophagy‐dependent ferroptosis.

Our results indicated that ferroptosis is closely associated with the skeletal muscle atrophy. The interaction between Nestin and LC3 is a crucial molecular event that antagonizes the autophagy system, prevents the degradation of autophagic ferritin, and hinders ferroptosis (Figure S10). Lindqvist et al. observed significant delays in healing in muscle deficient of nestin through muscle injury tests [14]. The H&E staining of the Nestin knockout mice clearly shown central nuclei, indicating active regeneration. Possibly, nestin deficiency rather destabilizes myocyte intermyofibrillar‐sarcolemnal connectivity, similar to dystrophin deficiency, thus making muscle more vulnerable to damage and causing multiple secondary effects. Therefore, the expression pattern of Nestin in myopathies such as DMD and the molecular regulatory mechanism of Nestin on Mdx mice can be further explored, providing potential targets for disease treatment and prevention.

## Conflicts of Interest

The authors declare no conflicts of interest.

## Supporting information


**Figure S1** **Ferroptosis occurs in skeletal muscle atrophy, and Nestin expression is decreased**. (A) Scheme of the Dex‐induced C2C12 myotubes atrophy model. And phase contrast images of C2C12 myotubes treated with Dex for 0, 24, 48, 72 h or Erastin for 48 h (*n* = 3). (B) Relative levels of Trim63 and MAFbx mRNA of expression of the indicated genes in myotubes after Dex treatment for the indicated times (*n* = 3). (C) Scheme of the tail suspension (TS) muscle atrophy model. Mice were suspended by their tails for 0, 3 or 7 d (TS) and compared with the mice freely moving on the ground (d0) (*n* = 6). And the relative muscle weight or average short diameter of muscle fibres in the gastrocnemius muscle following 0, 3 or 7 days following TS treatment (*n* = 6). (D) Relative mRNA expression levels of Trim63 and MAFbx were assessed at 0, 3 or 7 days following TS treatment (*n* = 3). (E) Relative mRNA and protein expression levels of Trim63, MAFbx, ACSL4, FTH1, and GPX4 were assessed. And the values of GSH, MDA, 4‐HNE and iron content were determined at 0, 3 or 7 days following TS treatment (*n* = 6). (F) qPCR and western blot analysis the expression of Nestin expression levels were assessed at 0, 3 or 7 days following TS treatment (*n* = 3). Data are means ± SD. One‐way ANOVA test was performed to compare multiple groups. *p < 0.05; **p < 0.01; ***p < 0.001.
**Figure S2. Nestin is highly expressed in muscles, and Nestin knockout induces skeletal muscle atrophy.** (A) Relative expression of Nestin mRNA levels in mouse tissues and cell (*n* = 6). (B) Targeting strategy for Nestin conditional knockout in mouse. (C) Real‐time PCR analysis of Nestin expression in mouse tissues from Nestin cKO mice and control mice in different organs or tissues. Skeletal muscle, Kidney, Liver, Lung, Spleen, Brain (*n* = 6). (D) Morphological aberrations in TA, soleus and EDL muscles were examined using H&E staining (*n* = 6). (E) Average myofiber size of muscle fibres were measured in TA, soleus and EDL from Nestin cKO mice and control mice (*n* = 6). (F) Body weight of male or female WT and Nes cKO mice was measured at 2 and 5 months (*n* = 6). Data are means ± SD. *p < 0.05; **p < 0.01; ***p < 0.001.
**Figure S3.** **Nestin could rescue skeletal muscle atrophy.** C2C12 myoblast cells were transfected with Nestin silenced and overexpression plasmid were expanded and induced to differentiate into myotubes in differentiation medium. (A) Relative expression levels of Nestin mRNA or protein levels in C2C12 cells at 48 h after transfection, control shRNA and pcDNA3.1 vector were used as control (*n* = 3). (B) Real‐time PCR analysis of Trim63 and MAFbx expression levels in C2C12 cells at 48 h after transfection, DMSO group was used as control (*n* = 3). (C) Western blot analysis of Trim63 and MAFbx proteins expression levels in C2C12 cells at 48 h after transfection (*n* = 3). (D) Myotubes were stained with anti‐myosin heavy chain (MyHC) antibody (red), and cell nuclei with DAPI (blue) in Nestin silenced or overexpression cells (*n* = 3). (E) Western blot analysis of Trim63 and MAFbx proteins expression levels in C2C12 cells after transfection, and then treatment with Dex for 24 h to induce myotubes atrophy (*n* = 3). (F) Immunofluorescence staining of MyHC to measure myotubes area in C2C12 cells after transfection, and then treatment with Dex for 24 h to induce myotubes atrophy (*n = 3*). Data are means ± SD. *p < 0.05; **p < 0.01; ***p < 0.001.
**Figure S4.** **Deletion of Nestin makes cells more susceptible to ferroptosis‐induced cell death.** C2C12 cells were treated with Erastin or RSL3 for 6 h, with or without the Liproxstatin‐1 at concentrations and time points. (A) CCK8 was used to detect cell viability at different concentrations of Liproxstatin‐1 following Erastin treatment (*n* = 6). (B) CCK8 was used to detect cell viability at different time points of Liproxstatin‐1 following Erastin treatment (*n* = 6). (C) CCK8 was used to detect cell viability at different concentrations of Liproxstatin‐1 following RSL3 treatment (*n* = 6). (D) CCK8 was used to detect cell viability at different time points of Liproxstatin‐1 following RSL3 treatment (*n* = 6). (E) CCK8 was used to detect cell viability in WT or Nes cKO cells treated with different concentrations of Erastin (*n* = 6). (F) PI staining was used to detect cell viability in WT or Nes cKO cells after treatment with Erastin (3 μM) for 12 h (*n* = 6). Data are means ± SD. *p < 0.05; **p < 0.01; ***p < 0.001.
**Figure S5. Liproxstatin‐1 alleviates myotube atrophy caused by Nestin knockout through the inhibition of ferroptosis.** (A) Nestin cKO myoblast cells were cultured in differentiation medium for 24 h, with or without Erastin or Lip‐1 for 24 h. CCK8 and PI staining were used to detect cell viability (*n* = 6). (B) ROS was detected by flow cytometry in Nestin cKO myoblast cells with or without Erastin or Lip‐1 for 24 h (*n* = 6). (C) Mitochondrial state was assessed in Nestin cKO myoblast cells using Mito‐Tracker Red CMXRos, with or without Erastin or Lip‐1 for 24 h. Scale bars, 50 μm (*n* = 6). (D) The values of intracellular GSH, MDA, 4‐HNE, iron content, and ROS levels were tested in Nestin cKO myoblast cells with or without Erastin or Lip‐1 for 24 h (n = 6). (E) Immunocytochemical staining of MyHC was performed using a pan‐myosin heavy chain antibody (Red) in Nestin cKO myoblast cells, with or without Erastin or Lip‐1 treatment for 24 h. DAPI was used to counterstain the nuclei (blue). Scale bars, 100 μm (*n* = 3). (F) The expression levels of Trim63 and MAFbx mRNA were analysed by qPCR in Nestin cKO myoblast cells, with or without Erastin or Lip‐1 treatment for 24 h (n = 3). Data are means ± SD. *p < 0.05; **p < 0.01; ***p < 0.001.
**Figure S6.** **Liproxstatin‐1 effectively inhibits ferroptosis and mitigates skeletal muscle atrophy after Nestin knockout.** Liproxstatin‐1 (5 mg/kg) was injected into the skeletal muscle of Nestin cKO mice for 4 weeks. (A) Western blot and qPCR analysis was used to measure the expression levels of ACSL4, FTH1, and GPX4 in Nestin cKO mice with or without injection of Liproxstatin‐1 (*n* = 3). (B) The values of GSH, MDA, 4‐HNE, and iron content were measured in Nestin cKO mice with or without injection of Liproxstatin‐1 (*n* = 6). (C) Representative graphs of GAS, SOL, EDL, and TA in Nestin cKO mice were generated with or without injection of Liproxstatin‐1 (*n* = 6). (D) The anti‐dystrophin antibody was used to stain the cross‐sectional area of the GAS muscle fibre. The relative average area is displayed on the right (*n* = 6). (E) Force measurements performed on GAS from Nestin cKO mice with or without injection of Liproxstatin‐1 (*n* = 6). (F) Western blot analysis was used to measure the expression of MAFbx and Trim63 protein in Nestin cKO mice with or without injection of Liproxstatin‐1 (*n* = 3). Data are means ± SD. *p < 0.05; **p < 0.01;
**Figure S7.** **Inhibition of autophagy by using the autophagy inhibitor CQ or knocking down ATG5 decreases the ferroptosis promoted by Nestin silenced.** (A) LC3B, Beclin1 and P62 protein expression were determined by western blot analysis in Nestin silenced and control cells after treated with CQ (20 μM) or DMSO for 24 h (*n* = 3). (B) LC3B, Beclin1 and P62 protein expression were determined by western blot analysis in Nestin silenced or control cells, with or without Ad‐shAtg5 cells for 24 h (*n* = 3). (C) The expression of ferroptosis‐associated proteins of ACSL4, FTH1 and GPX4 were determined by western blot analysis in Nestin silenced and control cells after treated with CQ for 24 h (*n* = 3). (D) The expression of ferroptosis‐associated proteins of ACSL4, FTH1 and GPX4 were determined by western blot analysis in Nestin silenced and control cells after treated or untreated with Ad‐shAtg5 cells for 24 h (*n* = 3). (E) GSH, MDA, 4‐HNE and iron content were measured in Nestin silenced and control cells after treated with CQ for 24 h (*n* = 6). (F) GSH, MDA, 4‐HNE and iron content were measured in Nestin silenced and control cells after treated or untreated with Ad‐shAtg5 cells for 24 h (*n* = 6). Data are means ± SD. *p < 0.05; **p < 0.01; ***p < 0.001.
**Figure S8.** **Nestin regulates LC3B at the protein level but not the mRNA level.** (A, B) Under Dex treatment (10 μM, 6 h), representative western blot and quantification of LC3B protein levels (*n* = 3). (C) LC3B mRNA expression was analysed by qPCR under Dex treatment (10 μM, 6 h) (*n* = 3). (D, E) Under Erastin treatment (5 μM, 6 h), representative western blot and quantification of LC3B protein levels (*n* = 3). (F) LC3B mRNA expression was analysed by qPCR under Erastin treatment (5 μM, 6 h) (*n* = 3). Data are means ± SD. *p < 0.05; **p < 0.01; ***p < 0.001.
**Figure S9.** **Inhibition of autophagy by Ad‐shLC3B decreases the ferroptosis promoted by Nestin silenced.** (A) Western blot analysis LC3B, Beclin 1 and P62 protein expression after transfected with either Ad‐shLC3B or Ad‐LC3B in Nestin silenced or control cells, then treated with Dex for 12 h (*n* = 3). (B) Detailed information on the experimental group in this part of the experiment. (C) GSH, MDA, 4‐HNE, and iron content were measured after transfected with either Ad‐shLC3B or Ad‐LC3B in Nestin silenced or control cells, then treated with Dex for 12 h (*n* = 6). (D) Western blot analysis the expression of ACSL4, FTH1 and GPX4 protein levels after transfection (*n* = 6). (E) PI staining and CCK8 were used to detect cell viability after transfection and different intervention conditions (*n* = 6). (F) The expression of Trim63 and MAFbx proteins expression levels was detected by western blotting after transfection (*n* = 3). Data are means ± SD. *p < 0.05; **p < 0.01; ***p < 0.001.
**Figure S10**. **Model of the role of Nestin in adult skeletal muscle atrophy.** Nestin ubiquitination LC3B antagonizes LC3‐mediated autophagy, thereby inhibiting ferroptosis signalling pathways to protect skeletal muscle atrophy.
Table S1. The primers used in this study.

## Data Availability

RNA‐seq data used in this investigation have been submitted to the Sequence Read Archive (SRA) at the National Center for Biotechnology Information with the accession code SUB9399493. All other data is contained in the article and its supplemental files or can be obtained from the authors upon request.
